# Laparoscopic repair of vesicovaginal fistulae with a transperitoneal approach at Universitas Gadjah Mada Urological Institute: a case report

This article has been retracted.

**DOI:** 10.1186/s13256-018-1582-6

**Published:** 2018-02-25

**Authors:** Indrawarman Soeroharjo, Said Alfin Khalilullah, Raden Danarto, Prahara Yuri

**Affiliations:** Division of Urology, Department of Surgery, Faculty of Medicine, Universitas Gadjah Mada/Dr. Sardjito Hospital, Yogyakarta, 55281 Indonesia

**Keywords:** Laparoscopic, Vesicovaginal fistulae, Urinary incontinence

## Abstract

**Background:**

A vesicovaginal fistula is an abnormal fistulous tract extending between the bladder and the vagina that allows the continuous involuntary discharge of urine into the vaginal vault. In addition, the sequelae from these fistulae have a profound effect on the patients in view of their physical, psychological, and social dimensions. The treatment of vesicovaginal fistula is surgical in most cases and the choice of the repair technique is controversial. We evaluated the benefits of a laparoscopic approach in a patient with vesicovaginal fistulae. Here, we present our first experience using a simplified laparoscopic approach technique to repair vesicovaginal fistulae in our country.

**Case presentation:**

A 46-year-old Javanese woman presented with urinary incontinence following an abdominal hysterectomy 3 months earlier and received laparoscopic repair. A cystoscopy was performed to confirm the fistula orifice and a stent was inserted into the fistula tract from her bladder to her vagina. A tamponade was inserted into her vagina up to the vaginal apex, to be able to identify the vagina. She had adhesions; therefore, adhesiolysis was performed using a combination of sharp and blunt dissection to expose the vaginal stump and the superior aspect of her bladder. A simple cystotomy was performed and extended to include the fistulae site, and then the defect was repaired by using a running stitch. A second layer of closure was performed in an imbricating fashion with the same suture. The vagina defect was not closed separately but covered with an omental flap. This procedure takes approximately 2.5 hours; estimated blood loss was minimal and there were no intraoperative complications. She had no recurrent symptoms 6 months after surgery.

**Conclusion:**

Our case report concludes that the simplified laparoscopic approach to vesicovaginal fistulae is a viable option for successful repair and that it reduces the size of bladder opening, causes minimal bleeding, and gives successful relief.

## Background

Vesicovaginal fistulae (VVF) represent a significant morbidity in female urology with an incidence that varies between 0.3 and 2%, most of which are iatrogenic [1]. It is estimated that 0.8 per 1000 of all hysterectomies are complicated by the development of a VVF. Other causes in the developed world include malignant disease and pelvic irradiation [2]. In contrast to obstetric and irradiation fistulas, the typical postsurgical (post-hysterectomy) fistula is the result of more direct and localized trauma to healthy tissue [3].

The success of VVF repair depends on various factors, including fistulae size, location, timing from the antecedent event, severity, quality of surrounding tissue, clinical experience, and surgical skill [1]. Surgical repairs of VVF are most commonly performed: (1) vaginally, (2) abdominally, and (3) laparoscopically. The approach to VVF repair is often dictated by surgeons’ preference and the location or complexity of the VVF. A surgeon’s preference is usually based on his or her training and experience [2].

Laparoscopic repair is now a well-established modality in the management of VVF, with a number of studies demonstrating its safety, feasibility, and efficacy with a good success rate and less morbidity compared with those of open surgery [1–3]. Our laparoscopic technique differs from other laparoscopic techniques; here, we report our first experience using laparoscopic approach for the management of VVF with decreasing laparoscopic intracorporeal suturing and highlight our results with this simplified laparoscopic approach.

## Case presentation

A 46-year-old Javanese woman presented with urinary incontinence following an abdominal hysterectomy with bilateral salpingectomy 3 months earlier. She is a housewife with no history of routine drug use and no prior history of hypertension, diabetes, allergies, or other chronic disease. She does not smoke tobacco and does not consume alcohol.

A physical examination revealed that her general condition was good and her vital signs were: blood pressure 112/74 mmHg, heart rate 89 beats per minute, respiratory rate 18 times per minute, and temperature 36.6 °C. There were no abnormalities in her chest and abdomen, or in musculoskeletal and neurological examinations. In a genitalia examination using a speculum, we identified fistulae above her vagina wall that were 1 cm in size. All laboratory findings (that is, complete blood count, liver functions, renal functions, and urine analysis) were within normal limits.

After discussion with our patient regarding the risks and benefits of an open abdominal procedure and laparoscopic approach, we discussed the similarities and differences between the two procedures were her. We chose surgical management using laparoscopic approach with the considerations that it could facilitate precise dissection, offer good visualization, and be minimally invasive, thereby enabling faster recovery.

### Surgical technique

Our patient was placed in the lithotomy position and received general anesthesia. A cystoscopy was performed to confirm the fistulae orifice and a stent was inserted into the fistulae tract from her bladder to her vagina. A tamponade was inserted into her vagina up to the vaginal apex, to be able to identify the vagina and prevent loss of pneumoperitoneum. A transperitoneal approach was performed with trocars distributed as follows: The camera was placed through a 12 mm port with 30° down lens located superior to the umbilicus. Two ports for the surgeon were placed on the right side (Fig. 1).

**Fig. 1:** Port placement for laparoscopic-assisted vesicovaginal fistulae repair. *A* assistant port, *C* camera port, *O* operator ports, *S* suction port

She had adhesions; therefore, adhesiolysis was performed, using a combination of sharp and blunt dissection to expose the vaginal stump and the superior aspect of her bladder (Fig. 2). A simple cystotomy was performed and extended to include the fistulae site, and the fistula tract was excised until viable fresh tissue was exposed. Later the defect was repaired by using a running stitch of 3–0 Vicryl. Knots were tied intracorporeally. A second layer of closure was performed in an imbricating fashion with the same suture. The vagina defect was not closed separately but covered with an omental flap (Fig. 3). A vascularized omental flap was made using a scalpel, which was placed in the plane of dissection between her bladder and her vagina, and it was secured with two attachment points.

**Fig. 2:** Sharp and blunt dissection to develop a separation plane between *A*, the anterior vaginal wall, and *B*, the posterior bladder wall surrounding the area of the fistulae

**Fig. 3:** **a** The vaginal defect was covered with an omental flap. **b** Cystorrhaphy with a braided suture in a vertical fashion. Note a suture above the bladder opening that was exteriorized to maintain countertraction

The ureteral stents were removed without difficulty. A urethral catheter was placed for adequate postoperative urinary drainage. This procedure takes approximately 2.5 hours; the estimated blood loss for our case was minimal and there were no intraoperative complications.

Our patient was given intravenously administered ceftriaxone 1 gram per 12 hours postoperatively for prophylaxis and orally administered diclofenac for pain control on an as-needed basis from the following day. At postoperative day 1, she was able to eat as usual and complained of minimal abdominal pain during mobilization. The surgical wound was good and there was no urine leakage from her vagina. After that, she was discharged while still using urethral catheter for adequate postoperative urine drainage for 2 weeks.

She returned for a follow-up 2 weeks after surgery and reported that she experienced no recurrent incontinence and urination was normal. She continued to do well at 1-month, 3-month, and 6-month postoperatively.

## Discussion

We present a case in which our patient underwent VVF repair for which a laparoscopic approach was used; there was no separate vaginal closure but the vaginal defect was covered with an omental flap and simple cystotomy, which may potentially reduce the recurrence rate and irritative voiding symptoms. Furthermore, the omental patch functions as a barrier and provides a robust blood supply and rich lymphatics to enhance tissue growth and maturation. This approach is an attractive alternative for managing VVF.

The laparoscopic approach in VVF has given new hope for the development of surgical techniques [4]. Most authors reported that with laparoscopy it is possible to achieve good illumination, magnification of vision, excellent exposure, direct and quick access to the fistulae, and high success rates, regardless of the technique used [2, 4–7]. Although the laparoscopic approach in expert hands may provide a high success rate, it is not widely practiced due to the costs and considerable learning curves imposed by intracorporeal laparoscopic suturing, a requirement for VVF repair, which is an advanced skill many surgeons lack [8, 9].

In this study, we reported a case of VVF repair using a simplified laparoscopic approach, which is effective because it quickly locates the fistulae, reduces the size of the bladder opening, shortens operative times, decreases irritative symptoms, and minimizes the risk of dehiscence and leakage [8]. Two modifications constituted the simplified laparoscopic approach: (1) simple cystotomy and (2) no separate vaginal closure. The simple cystotomy approach provides adequate visualization while at the same time minimizing the complications of the standard O’Conor cystotomy.

The simple cystotomy approach has been previously described as Mini O’Conor vesicotomy [8]. The classical O’Conor technique involves a large cystotomy, which starts at the bladder dome and extends down the posterior bladder wall to the site of the fistula, thus bivalving the bladder. It increases the complexity of subsequent laparoscopic suturing and adds significantly to operative duration and possibly also contributes to bladder spasms in the postoperative period.

The aims of the technique of closure of the bladder without separate closure of the vaginal opening and covering the vaginal opening with an omental flap are to enhance blood supply, protect suture line, and close dead space. The omental patch functions as a barrier and provides blood supply and rich lymphatics to enhance tissue growth and maturation.

The best way for a surgeon to achieve successful repair is by using the type of surgery with which he or she is most familiar. Techniques of repair include: (1) the vaginal approach, (2) the abdominal approach, and (3) the laparoscopic approach [2, 3]. The literature documents excellent success rates for the treatment of VVF if the following general surgical principles are followed: (a) careful evaluation of the type of fistulae, (b) watertight bladder closure without tension, (c) suture on healthy tissues with good blood supply and without the presence of infection, and (d) adequate postoperative urine drainage [10, 11].

Only a few studies have compared the surgical approach for patients with VVF [6, 12–14]. Several studies have published that there is no difference between surgical outcome and complication rates between open and laparoscopic approaches [13, 14]. Phsak *et al*. compared the outcome between recurrent VVF and primary VVF without tissue interposition [13]; they concluded that transvaginal approach of recurrent VVF without tissue interposition is as equally successful as primary repairs [13]. Also, Rajamaheswari *et al*. reported the outcome between a vaginal and transabdominal approach and they found a comparable success rate between the two groups [14]. In contrast, another study compared the surgical procedure between laparoscopic-open abdominal-transvaginal in patients with VVF. Their data found that laparoscopic approach had a better outcome and lower morbidity than transabdominal and vaginal approaches [6].

The right time for surgery in patients with VVF is still unclear. One study by Blaivas *et al*. [15] concluded that early repair of the VVF has the advantage of shortening period of discomfort for the patient. However, delayed surgical repair of the VVF may be accepted if the underlying disease leads to an inflammatory process such as after radiotherapy or obstetric trauma [2, 10]. Contrary to these statements, delayed surgery was performed in this study.

One retrospective chart review by Javali *et al*. [16] with a total of 22 patients on whom a laparoscopic approach to VVF repair was performed produced excellent results with minimal morbidity. All patients were continent after catheter removal at postoperative day 14 and remained symptom free in the follow-up period, which ranged from 2 to 45 months. They also reported no open conversions and no intraoperative complications with minimal estimated blood loss.

As with the above study [16], our study also found no intraoperative complications and no recurrent incontinence had been experienced at the 6-month follow-up. According to this, we think that the laparoscopic approach could be adopted in our country to repair VVF with excellent results.

There are two approaches to repair VVF laparoscopically: single or double layers of bladder closure with or without tissue interposition. Most of the literature summarizes that the same results are obtained using either of these approaches [2]. Although our study used double layers of bladder closure with tissue interposition and showed a good outcome, it is difficult to conclude that other techniques do not produce good outcomes. From one meta-analysis study, the surgical techniques of single or double layer bladder closure and interposition showed no statistical differences [2, 6] Therefore, the decision to choose a particular technique of layers of closure and interposition graft remains controversial and is a personal decision based on a surgeon’s experience.

## Conclusions

In the current report we have described our first experience using a simplified laparoscopic approach for the treatment of VVF. Successful treatment using a laparoscopic approach in VVF is highly dependent on the surgeon’s experience, tissue conditions around fistulae, tension-free watertight closure, and adequate postoperative urinary drainage. A VVF treated with simplified laparoscopic approach of simple cystotomy and no separate vaginal closure in our study was successfully relieved without recurrent symptoms. Additional studies with a large number of cases and comparison of these techniques with other approaches are required.

## Abbreviation

VVF: Vesicovaginal fistulae
